# Effects of Ginsenoside Rg1 on the Biological Behavior of Human Amnion-Derived Mesenchymal Stem/Stromal Cells (hAD-MSCs)

**DOI:** 10.1155/2023/7074703

**Published:** 2023-02-15

**Authors:** Li Ling, Han Shu, Yubin Huang, Jiying Hou, Yuanyuan Hua

**Affiliations:** ^1^Department of Obstetrics and Gynecology, The Second Affiliated Hospital of Chongqing Medical University, Chongqing 400010, China; ^2^Department of Histology and Embryology, Laboratory of Stem Cell and Tissue Engineering, Chongqing Medical University, Chongqing 400010, China

## Abstract

Ginsenoside Rg1 (Rg1) is purified from ginseng with various pharmacological effects, which might facilitate the biological behavior of human amnion-derived mesenchymal stem/stromal cells (hAD-MSCs). This study is aimed at investigating the effects of Rg1 on the biological behavior, such as viability, proliferation, apoptosis, senescence, migration, and paracrine, of hAD-MSCs. hAD-MSCs were isolated from human amnions. The effects of Rg1 on the viability, proliferation, apoptosis, senescence, migration, and paracrine of hAD-MSCs were detected by CCK-8, EdU, flow cytometry, SA-*β*-Gal staining, wound healing, and ELISA assays, respectively. The protein expression levels were detected by western blot. Cell cycle distribution was evaluated using flow cytometry. We found that Rg1 promoted hAD-MSC cycle progression from G0/G1 to S and G2/M phases and significantly increased hAD-MSC proliferation rate. Rg1 activated PI3K/AKT signaling pathway and significantly upregulated the expressions of cyclin D, cyclin E, CDK4, and CDK2 in hAD-MSCs. Inhibition of PI3K/AKT signaling significantly downregulated the expressions of cyclin D, cyclin E, CDK4, and CDK2, prevented cell cycle progression, and reduced hAD-MSC proliferation induced by Rg1. hAD-MSC senescence rate was significantly increased by D-galactose, while the elevated hAD-MSC senescence rate induced by D-galactose was significantly decreased by Rg1 treatment. D-galactose significantly induced the expressions of senescence markers, p16^INK4a^, p14^ARF^, p21^CIP1^, and p53 in hAD-MSCs, while Rg1 significantly reduced the expressions of those markers induced by D-galactose in hAD-MSCs. Rg1 significantly promoted the secretion of IGF-I in hAD-MSCs. Rg1 reduced the hAD-MSC apoptosis rate. However, the difference was not significant. Rg1 had no influence on hAD-MSC migration. Altogether, our results demonstrate that Rg1 can promote the viability, proliferation, and paracrine and relieve the senescence of hAD-MSCs. PI3K/AKT signaling pathway is involved in the promotive effect of Rg1 on hAD-MSC proliferation. The protective effect of Rg1 on hAD-MSC senescence may be achieved via the downregulation of p16^INK4A^ and p53/p21^CIP1^ pathway.

## 1. Introduction

Mesenchymal stem cells (MSCs) are a kind of multipotent adult stem cells which show the ability in self-renewal, multilineage differentiation, immune modulation, proangiogenesis, and anti-inflammation [1, 2]. MSCs can be isolated from a broad subset of tissue sources, such as amniotic membrane, amniotic fluid, umbilical cord, bone marrow, dental pulp, and adipose tissue [1, 2]. In previous studies, MSCs have been explored to treat various diseases [3, 4]. Recently, MSC transplantation has become a promising and focal treatment for the regeneration of injured tissue and refractory diseases [1, 4, 5].

Besides the features of MSCs, human amnion-derived mesenchymal stem/stromal cells (hAD-MSCs) have been proved to have some other advantages such as relative high proliferation rates, multidifferentiation potential, low/no immunogenicity, no tumorigenicity, no ethical or legal concerns, and noninvasive acquisition process [6–9]. Amniotic membranes are a rich cellular source of MSCs, and approximately 2 × 10^6^ of hAD-MSCs are available for use at 3 days after the primary isolation and culture of 1 g of amniotic tissue samples [9]. These advantages make hAD-MSCs a promising source of stem cells for tissue engineering and regenerative medicine.

During the expansion of MSCs *in vitro*, there are some uncontrolled factors, such as the limited number of primary MSCs [2, 10], the decreases of proliferation and differentiation capacity of MSCs after passaging, and the interdonor variability and scalability associated with primary donor-derived MSCs [4, 11, 12], which may affect the number and quality of MSCs before clinical utility [1, 2, 13]. During the transplantation of MSCs, there are still various unsolved problems, such as the loss of MSCs, low homing and engraftment rates of MSCs, inability of precise regulation of MSC differentiation, and accelerated senescence and apoptosis of MSCs after cell transplantation, which are major issues in MSC preclinical research and may influence the clinical utility of MSCs [1–3]. Thus, it is imperative to solve the issues mentioned above and optimize the biological behavior of MSCs for the improvement of the therapeutic efficacy of MSC transplantation for various diseases.

Ginsenoside Rg1 (Rg1) is purified from the stem or root of ginseng with various pharmacological effects such as antiaging, anti-inflammatory, and antioxidant properties [14–16]. Rg1 regulates organ function in the human body, which is inseparable from its regulation of adult stem cells [2]. Bone marrow-derived mesenchymal stem cells (BM-MSCs) are a traditional source of MSCs [17], which are most widely researched in cell-based therapy [18]. However, the acquisition process of BM-MSCs is invasive and the number of BM-MSCs isolated from bone marrow is less [19]. In addition, the number and function of BM-MSCs will reduce accompanied with the increase of the donor's age [20–22]. These issues may influence the utility of BM-MSCs in cell-based therapy. Some studies have found that Rg1 might effectively regulate the proliferation, differentiation, apoptosis, senescence, and paracrine of BM-MSCs [23–27]. However, the effects of Rg1 on the biological behavior of hAD-MSCs, a promising seed cell in tissue engineering, are still unknown.

In this study, the effects of Rg1 on the biological behavior, such as viability, proliferation, apoptosis, senescence, migration, and paracrine, of hAD-MSCs were investigated. Rg1 might provide a promising application prospect with regard to the regulation of hAD-MSCs to promote the therapeutic efficacy of hAD-MSC transplantation for diseases.

## 2. Materials and Methods

The research was in compliance with the Helsinki Declaration and approved by the Ethics Committee of the Second Affiliated Hospital of Chongqing Medical University (permit number 2020-20).

### 2.1. Reagents

Rg1 (molecular formula: C42H72O14) was purchased from Yuanye Bio-Technology Co., Ltd. (Shanghai, China). Fetal bovine serum (FBS), Dulbecco's modified eagle medium low-glucose (L-DMEM), and 0.05% trypsin and 0.02% ethylenediaminetetraacetic acid (EDTA) were purchased from Gibco Co. (Grand Island, NY, USA). Collagenase II was purchased from Sigma-Aldrich (St. Louis, MO, USA). DNase I was purchased from Worthington Biochemical Co. (Lakewood, New Jersey, USA). 5-ethynyl-2′-deoxyuridine (EdU) was purchased from RiboBio Co., Ltd. (Guangzhou, China). D-galactose (D-gal) was purchased from Macklin Biochemical Co., Ltd. (Shanghai, China). Enzyme-linked immunosorbent assay (ELISA) kit for insulin-like growth factor-I (IGF-I) was purchased from Uscn Life Science (Wuhan, Hubei, China). Cyclin D1, cyclin E1, cyclin-dependent kinase 2 (CDK2), cyclin-dependent kinase 4 (CDK4), p21^CIP1^, and p53 antibodies were purchased from Proteintech Group, Inc. (Wuhan, China). Protein kinase B (Akt), phospho-Akt, p14^ARF^, and p16^INK4a^ antibodies were purchased from Affinity Biosciences (Jiangsu, China). ReverTra Ace-*α*-first strand cDNA Synthesis Kit was purchased from TOYOBO Life Science (Shanghai, China). TRIzol Reagent was purchased from Invitrogen of Thermo Fisher Scientific (Carlsbad, CA, USA). Chondrogenic, adipogenic, and osteogenic differentiation medium, alizarin red S, alcian blue, and oil red O were purchased from Cyagen Biosciences Inc. (Suzhou, China). All other chemicals were purchased from Beyotime Institute of Biotechnology (Haimen, China).

### 2.2. Isolation, Culture, and Identification of hAD-MSCs

Primary hAD-MSCs were isolated, cultured, and identified according to our previous published research [4, 17]. Donors (*n* = 18) were healthy full-term pregnant women from the Second Affiliated Hospital of Chongqing Medical University, China. They received cesarean sections, and their placentas were collected after writing informed consent. Amnions were separated from term placentas and digested with 0.05% trypsin and 0.02% EDTA for 40 min at 37°C. After the filtration by a 300-mesh sieve, the residue tissue was collected. Then, the above process was repeated. After that, the residue tissue was digested with 0.75 mg/mL collagenase II in combination with 0.075 mg/mL DNase I at 37°C for 1.5 h. After the filtration by a 300-mesh sieve, the cells were collected by the centrifugation of filter liquor at 1500 r/min for 10 min. The isolated cells were cultured in the L-DMEM medium at a density of 5 × 10^5^ cells/cm^2^, supplemented with 12% FBS, 0.1 mg/mL streptomycin, and 100 U/mL penicillin, in a humidified atmosphere with 5% CO_2_ at 37°C. When 90–100% of cell confluency was reached, cells were passaged at a ratio of 1 : 2.

The third passage of isolated cells was used for identification, which was published in our previous studies [17]. An inverted microscope (Olympus Corporation, Tokyo, Japan) was used to observe the morphological characteristics of isolated cells. Flow cytometry was used to detect the expression of surface markers of MSCs on isolated cells. For the identification of multipotent differentiation, isolated cells were cultured in chondrogenic, adipogenic, or osteogenic differentiation medium at a density of 1 × 10^5^ cells/cm^2^ for 21 days. Then, cells were stained with alcian blue, oil red O, or alizarin red S and observed under the inverted microscope.

The third passage of hAD-MSCs was used for the subsequent experiments.

### 2.3. Ginsenoside Rg1 Preparation and Optimization Concentration of Rg1 Treatment

Rg1 was dissolved in dimethylsulfoxide (DMSO) solution with high concentration for storage and then diluted with L-DMEM for use [28]. hAD-MSCs were exposed to Rg1 in the Rg1 group, while hAD-MSCs received pseudotreatment (without Rg1) in the control group. The optimal concentration of Rg1 was determined by Cell Counting Kit-8 (CCK-8) assay as follows.

### 2.4. CCK-8 Assay

CCK-8 assay was used to detect cell viability according to the manufacturer's instructions. hAD-MSCs were seeded at a concentration of 5 × 10^4^ cells/mL, cultured for 2 h, and exposed to different concentrations of Rg1 (0, 10, 20, 30, or 40 *μ*g/mL) or D-gal (0, 5, 10, 20, or 40 mg/mL) in 96-well plates. Then, the optical density (OD) value of cells was detected at 24 and 48 h after treatment for concentration optimization or at 24, 48, 72, 96, and 120 h after treatment for growth curves, at 450 nm using a plate reader (1510 model; Thermo Fisher Scientific Oy, Vantaa, Finland).

To explore the effect of phosphatidylinositol-3-kinase (PI3K)/AKT signaling on the proliferation of hAD-MSCs induced by Rg1, hAD-MSCs were cultured for 24 h and pretreated with or without LY294002 for 1 h followed by the treatment with or without Rg1 in the control, Rg1, Rg1+LY294002, and LY294002 groups. At 24 h after treatment, the OD value was measured.

### 2.5. Flow Cytometry

hAD-MSCs were cultured at a concentration of 1 × 10^5^ cells/mL in six-well plates.

For cell cycle assay, cells were cultured for 24 h and starved in serum-free mediums for 12 h. After that, hAD-MSCs were pretreated with LY294002 at a concentration of 50 *μ*mol/L for 1 hour as inhibitor treatment. Then, serum-free mediums were replaced with complete mediums with or without Rg1. At 24 h after treatment, hAD-MSCs (1 × 10^6^ cells/per tube) were fixed with precooled ethanol at a concentration of 70% and then incubated with propidium iodide (PI) and RNase A. The cell cycle was detected at 488 nm of excitation wavelength by a FACSCalibur flow cytometer (BD Biosciences).

For cell apoptosis assay, cells were divided into the control, Rg1, D-gal, and Rg1+D-gal groups. hAD-MSCs were treated with solvent or D-gal (40 mg/mL) for 24 h. Then, mediums were replaced with complete mediums with or without Rg1 (10 *μ*g/mL). After 24 h, cells were collected (1 × 10^6^ cells/per tube) and incubated with annexin-V-fluorescein isothiocyanate (FITC) and PI. Then, flow cytometry was used to detect the hAD-MSC apoptosis rate.

### 2.6. EdU Assay

hAD-MSCs were seeded in 24-well plates at a concentration of 1 × 10^5^ cells/mL, cultured for 24 h, and exposed to solvent or Rg1 (10 *μ*g/mL). hAD-MSCs were pretreated with LY294002 at a concentration of 50 *μ*mol/L for 1 hour as inhibitor treatment. At 24 h after Rg1 treatment, hAD-MSC proliferation was detected by EdU assay according to the manufacturer's instructions. Then, cells were observed under a fluorescent microscope (Nikon Corporation, Tokyo, Japan) or a laser scanning confocal microscope (Nikon Corporation, Tokyo, Japan). Image-Pro Plus 6.0 software (Media Cybernetics, Bethesda, MD, USA) was used to count Hoechst33342 and EdU positive cells. hAD-MSC proliferation rate was defined as EdU positive cells (red cells)/Hoechst33342 positive cells (blue cells) [4].

### 2.7. Aging-Related *β*-Galactosidase (SA-*β*-Gal) Staining

Cells were treated as described in apoptosis assay. Senescent cells were detected by SA-*β*-Gal staining kit according to the manufacturer's instructions, which were stained blue. Cells were randomly observed and counted in 200× microscopic fields under an inverted microscope [4]. The hAD-MSC senescence rate was defined as SA-*β*-Gal positive cells (blue cells)/total cells [4].

### 2.8. Western Blot

To explore the mechanisms of Rg1 on the senescence of hAD-MSCs, cells were treated as described in apoptosis assay. To explore the mechanisms of Rg1 on the proliferation of hAD-MSCs, hAD-MSCs were cultured for 24 h and starved in serum-free mediums for 12 h. Then, hAD-MSCs were pretreated with or without LY294002 for 1 h at a concentration of 50 *μ*mol/L followed by the treatment with or without Rg1 (10 *μ*g/mL). At 24 h after treatment, RIPA lysis buffer was used to treat hAD-MSCs, and the proteins in hAD-MSCs were extracted after centrifugation. The isolated proteins were quantified using Bradford Protein Assay Kit, separated by sodium dodecyl sulfate polyacrylamide gel electrophoresis (SDS-PAGE), and electrotransferred to polyvinylidene difluoride (PVDF) membranes (Millipore, USA). The membranes were washed, blocked, incubated with the specific primary antibodies of Akt (1 : 1000 dilution, AF6261), phospho-Akt (Ser 473, 1 : 1000 dilution, AF0016), cyclin D1 (1 : 10000 dilution, 26939-1-AP), cyclin E1 (1 : 1000 dilution, 11554-1-AP), CDK2 (1 : 5000 dilution, 10122-1-AP), CDK4 (1 : 2000 dilution, 11026-1-AP), p14^ARF^ (1 : 2000 dilution, AF0229), p21^CIP1^ (1 : 2000 dilution, 10355-1-AP), p53 (1 : 1000 dilution, 21891-1-AP), or p16^INK4a^ (1 : 1000 dilution, BF0580), and then incubated with the corresponding secondary antibodies (horseradish peroxidase-conjugated, 1: 2000 dilution, A0208, or A0216). Color development was processed using BeyoECL Plus kit according to the manufacturer's instructions.

### 2.9. Wound Healing Assay

Wound healing assay was performed to detect hAD-MSC migration. hAD-MSCs were seeded in 6-well plates at a concentration of 1 × 10^5^ cells/mL and cultured to 100% confluence. Then, a 200 *μ*L pipette tip was used to scratch wounds among the area of hAD-MSCs in the 6-well plates (3 wounds per well) [4]. After treatment, the medium was replaced with new medium containing only 2% of FBS. After that, hAD-MSCs were treated with and without Rg1 (10 *μ*g/mL) in the Rg1 and control groups, respectively. The scratched and covered areas were imaged at 0, 12, and 24 h after scratch under an inverted microscope. The area of scratch was measured by ImageJ v1.42q software (National Institutes of Health, USA). Covered area/scratched area × 100%, which was defined as the area-covered ratio of migration cells (ACRMC), was counted [4].

### 2.10. Real-Time Quantitative Polymerase Chain Reaction (RT-qPCR)

Cells were cultured at a concentration of 1 × 10^5^ cells/mL in 6-well plates for 24 h and exposed to Rg1 solution or solvent (an equivalent volume of DMSO diluted in L-DMEM) for 24 h. The contents in Table 1 showed the primers used in this experiment. *β*-Actin was chosen as the internal reference. RNA samples were extracted using TRIzol Reagent. The extracted RNA samples were quantified and then reversely transcribed into cDNA. A CFX96 Real-Time PCR Detection System (Bio-Rad, Hercules, CA, USA) with SYBR Green Real-Time PCR Master Mix (TOYOBO Life Science) was used to perform RT-qPCR. Target gene expression was confirmed using the 2^−ΔΔCt^ method.

### 2.11. ELISA

hAD-MSCs were cultured at a concentration of 1 × 10^5^ cells/mL in 6-well plates for 24 h and then exposed to Rg1 or solvent for 5 days. After that, the hAD-MSC supernatant was collected for the detection of IGF-I level according to the manufacturer's instructions.

### 2.12. Statistical Analysis

Statistical analyses were processed by SPSS 22.0 software (IBM, NY, USA). At least three independent experiments were performed in this study for all assays. Data was presented in the form of means ± standard deviations (SD). The independent sample *t-*test was used for two-group comparison, while one-way analysis of variance (ANOVA) was used for multiple-group comparison. Statistical significance was set to *P* < 0.05.

## 3. Results

### 3.1. Determination of the Optimal Concentration of Ginsenoside Rg1 on hAD-MSCs

The isolated cells grew as adherent cultures and displayed a fibroblastic morphology (Figures 1(a)–1(c)). The isolated cells were certified to have the ability to differentiate into osteoblasts, adipocytes, and chondroblasts under standard differentiating conditions *in vitro* (Figures 1(d)–1(l)). These cells have been identified as hAD-MSCs by our previous published studies [4, 17], which also have the common characteristics of MSCs [4, 17].

To explore the effects of Rg1 (Figure 1(p), image from PubChem) with different concentrations on the hAD-MSC viability, CCK-8 assay was performed. Our results found that the mean OD values of the Rg1 groups (10, 20, 30, and 40 *μ*g/mL of Rg1) were significantly higher than those of the control group (0 *μ*g/mL of Rg1) from 24 to 48 h (*P* < 0.01, Figure 1(q)). However, there was no significant difference between those Rg1 groups. Compared to the control group, Rg1 with the concentrations from 10 *μ*g/mL to 40 *μ*g/mL significantly promoted the viability of hAD-MSCs in the Rg1 groups (*P* < 0.01, Figure 1(q)). Thus, the minimum effective concentration of Rg1, 10 *μ*g/mL, was selected for the subsequent experiments.

### 3.2. Effects of Ginsenoside Rg1 on the Proliferation of hAD-MSCs

Cell cycle distribution of hAD-MSCs in the Rg1 and control groups was analyzed by flow cytometry. We found that, compared to the control group, the distribution of hAD-MSCs in G0/G1 phase after Rg1 treatment significantly decreased, while the distribution of hAD-MSCs in S and G2/M phases significantly increased, in the Rg1 group (*P* < 0.01, Figures 2(a) and 2(b)). These results demonstrate that Rg1 may promote cell cycle progression and might facilitate the proliferation of hAD-MSCs.

To define the effects of Rg1 on the proliferation of hAD-MSCs, a sensitive and specific method, EdU incorporation assay, was performed. We found that the hAD-MSC proliferation rate of the control group was significantly lower than that of the Rg1 group (*P* < 0.05, Figures 2(c) and 2(d)). The growth curves of hAD-MSCs were also investigated by CCK-8 assay in the Rg1 and control groups. Our results found that Rg1 significantly promoted the growth of hAD-MSCs (*P* < 0.01, Figure 2(e)). These results demonstrate that Rg1 can promote the proliferation of hAD-MSCs.

Cell proliferation is the process whereby cells reproduce themselves by growing and then dividing into two equal copies. As the cell cycle gradually enters S and G2/M phases from G0/G1 phase, cell proliferation is finally fulfilled. G1/S transition is essential for cell cycle progression [29]. Towards the end of G1, there is a restriction point, which marks the point where the cell becomes irreversibly committed to traverse the rest of the cell cycle [29]. It is known that cell cycle progression is regulated by the continuous activation of CDKs and cyclins [30]. The G1-to-S-phase transition is regulated by cyclin D/CDK4 and cyclin E/CDK2 during the cell cycle [31]. Thus, to explore the mechanisms of Rg1 on the cell cycle progression and proliferation of hAD-MSCs, the expressions of cyclin D, cyclin E, CDK4, and CDK2 in hAD-MSCs were detected by western blot in the Rg1 and control groups. Our results showed that the expressions of cyclin D1, CDK4, cyclin E1, and CDK2 in the Rg1 group were significantly higher than those in the control group (*P* < 0.05, Figures 3(a) and 3(b)). These results demonstrate that Rg1 can upregulate the expressions of cyclins and CDKs, which may result in cell cycle progression and proliferation of hAD-MSCs.

PI3K/Akt signaling is an important pathway which regulates cell cycle progression and boosts cell proliferation and survival [32, 33]. Our previous studies have also demonstrated that PI3K/Akt signaling pathway might play an important role in the proliferation of hAD-MSCs [17]. To further explore the upstream signaling of cyclins and CDKs for the mediation of Rg1-induced hAD-MSC proliferation, the key proteins of the PI3K/Akt signaling pathway were detected by western blot. It was found that the level of phospho-Akt was significantly increased by Rg1 treatment in hAD-MSCs (*P* < 0.01, Figures 3(a) and 3(b)). These results demonstrate that Rg1 can promote the phosphorylation of Akt and activate PI3K/Akt signaling pathway in hAD-MSCs.

To confirm whether PI3K/Akt pathway is the upstream signaling of cyclins and CDKs for the mediation of Rg1-induced hAD-MSC proliferation, the effects of PI3K/AKT signaling on the expression of regulatory proteins of cell cycle in Rg1-induced hAD-MSCs were detected. The results showed that, compared to the control group, the expression levels of cyclin D, cyclin E, CDK4, and CDK2 were significantly increased in hAD-MSCs after Rg1 treatment in the Rg1 group (*P* < 0.05, Figures 3(a) and 3(b)), while compared to the Rg1 group, inhibitor LY294002 pretreatment significantly inhibited the expression of phospho-Akt and reduced the elevated expression levels of cyclin D, cyclin E, CDK4 and CDK2 induced by Rg1 in hAD-MSCs in the Rg1+LY294002 group (*P* < 0.01, Figures 3(a) and 3(b)). The results demonstrate that Rg1 can activate PI3K/AKT signaling pathway, and inhibition of PI3K/AKT signaling influences the expression of regulatory proteins of cell cycle in Rg1-induced hAD-MSCs. The expressions of CDKs and cyclins might be downstream molecules regulated by PI3K/AKT signaling pathway in Rg1-induced proliferation of hAD-MSCs.

To further confirm the effect of PI3K/AKT signaling on the cell cycle progression and proliferation of hAD-MSCs mediated by Rg1, hAD-MSCs were pretreated with the PI3K/AKT signaling inhibitor, LY294002, before Rg1 treatment. Our results found that, compared to the control group, the distribution of cells in G0/G1 phase was significantly decreased, while the distribution of cells in S and G2/M phases was significantly increased in hAD-MSCs after Rg1 treatment in the Rg1 group (*P* < 0.01, Figures 4(a) and 4(b)). Compared to the Rg1 group, the distribution of cells in G0/G1 phase was significantly increased, while the distribution of cells in S and G2/M phases was significantly decreased by LY294002 pretreatment before Rg1 treatment in hAD-MSCs in the Rg1+LY294002 group (*P* < 0.01, Figures 4(a) and 4(b)). These results demonstrate that Rg1 can promote cell cycle progression of hAD-MSCs, and inhibition of PI3K/AKT signaling can prevent the cell cycle progression from G0/G1 phase into S and G2/M phases in Rg1-induced hAD-MSCs.

The CCK-8 assay showed that hAD-MSC viability and proliferation of the Rg1 group were significantly higher than those of the Rg1+LY294002 and control groups, while hAD-MSC viability and proliferation of the Rg1+LY294002 group were significantly lower than those of the control group at 24 h after Rg1 treatment (*P* < 0.01, Figure 4(c)). The EdU assay also showed that the hAD-MSC proliferation rate of the Rg1 group was significantly higher than that of the Rg1+LY294002 and control groups, while the hAD-MSC proliferation rate of the Rg1+LY294002 group was significantly lower than that of the control group at 24 h after Rg1 treatment (*P* < 0.01, Figures 4(d) and 4(e)). The results presented above prove that PI3K/AKT signaling pathway is involved in the promotive effect of Rg1 on hAD-MSC proliferation.

To sum up, the above results demonstrate that Rg1 may induce cell cycle progression and further promote the proliferation of hAD-MSCs through the upregulation of the expressions of CDKs and cyclins in hAD-MSCs. PI3K/Akt signaling pathway may be the upstream signaling of cyclins and CDKs for the mediation of Rg1-induced hAD-MSC proliferation.

### 3.3. Effects of Ginsenoside Rg1 on the Apoptosis of hAD-MSCs

To determine whether Rg1 affects hAD-MSC apoptosis, cell apoptosis rates were detected by flow cytometry. The results showed that Rg1 had no influence on the morphology of hAD-MSCs (Figure 5(b)). The hAD-MSC apoptosis rate of the Rg1 group was lower than that of the control group (Figures 5(c) and 5(d)). However, the difference was not significant between them (*P* > 0.05, Figures 5(c) and 5(d)).

To further confirm the effects of Rg1 on the apoptosis of aging hAD-MSCs, D-gal was used to establish the aging models of hAD-MSCs *in vitro*. The results showed that D-gal at the concentration of 40 mg/mL significantly inhibited the viability of hAD-MSCs at 24 and 48 h after D-gal treatment (*P* < 0.01, Figure 5(a)), which was selected for the subsequent experiments. The results further showed that D-gal inhibited the growth of hAD-MSCs (Figure 5(b)). Compared to the control group, D-gal significantly induced the apoptosis of hAD-MSCs in the D-gal group (*P* < 0.01, Figures 5(c) and 5(d)). The hAD-MSC apoptosis rate of the Rg1+D-gal group was lower than that of the D-gal group (Figures 5(c) and 5(d)). However, the difference was also not significant between them (*P* > 0.05, Figures 5(c) and 5(d)).

These results demonstrate that although Rg1 can inhibit the apoptosis of hAD-MSCs to some extent, the difference is not significant.

### 3.4. Effects of Ginsenoside Rg1 on the Senescence of hAD-MSCs

To explore the effects of Rg1 on the senescence of hAD-MSCs, senescent cells were detected by SA-*β*-Gal staining. D-gal was used to establish hAD-MSC aging models *in vitro*. It was found that D-gal significantly induced the senescence of hAD-MSCs (*P* < 0.01, Figures 6(a) and 6(b)). Compared to the control group, the hAD-MSC senescence rate significantly increased in the D-gal group (*P* < 0.01, Figures 6(a) and 6(b)). Compared to the D-gal group, the hAD-MSC senescence rate significantly decreased in the Rg1+D-gal group (*P* < 0.01, Figures 6(a) and 6(b)).

The senescent state is primarily characterized by durable cell cycle arrest [34]. DNA damage is an important mechanism of MSC senescence. DNA damage response is triggered by exogenous and endogenous stresses, resulting in the activation of two main senescence-related signaling pathways, p16^INK4A^ and p53/p21^CIP1^, which leads to cell cycle arrest and MSC senescence [34]. To further explore the mechanisms of Rg1 on the senescence of hAD-MSCs, the expressions of relevant proteins of cell senescence and regulatory proteins of cell cycle were detected by western blot. It was found that, compared to the control group, the expressions of senescence markers, p16^INK4a^, p14^ARF^, p21^CIP1^, and p53, were significantly increased, while the expressions of cyclin D1, cyclin E1, and CDK4 were significantly decreased in hAD-MSCs after D-gal treatment in the D-gal group (*P* < 0.05, Figures 6(c) and 6(d)). Compared to the D-gal group, the expressions of p16^INK4a^, p14^ARF^, p21^CIP1^, and p53 were significantly decreased, while the expressions of cyclin D1, cyclin E1, and CDK4 were significantly increased by Rg1 treatment in hAD-MSCs in the Rg1+D-gal group (*P* < 0.01, Figures 6(c) and 6(d)).

These results demonstrate that Rg1 can downregulate p16^INK4A^ and p53/p21^CIP1^ pathways and relieve the senescence of hAD-MSCs.

### 3.5. Effects of Ginsenoside Rg1 on the Migration of hAD-MSCs

To explore the effects of Rg1 on the migration of hAD-MSCs, wound healing assay was performed. At 0 h after scratch, there was no significant difference in the scratched area between the control and Rg1 groups (Figure 7(a)). At 12 and 24 h after scratch, there was also no significant difference in the ACRMC between the control and Rg1 groups (*P* > 0.05, Figures 7(a) and 7(b)). These results demonstrate that Rg1 might have no influence on the migration of hAD-MSCs *in vitro*.

### 3.6. Effects of Ginsenoside Rg1 on the Paracrine of hAD-MSCs

To explore the effects of Rg1 on the paracrine of hAD-MSCs, RT-qPCR was performed to detect the expressions of cytokines secreted by MSCs which have been reported [7, 35]. It was found that the relative mRNA expression level of IGF-I in hAD-MSCs was significantly higher in the Rg1 group than in the control group (*P* < 0.01, Figure 8(e)). Compared to the control group, the relative mRNA expression levels of interleukin- (IL-) 10 and hepatocyte growth factor (HGF) were higher (Figures 8(a)–8(f)), while the relative mRNA expression levels of IL-1*β*, IL-6, granulocyte-colony-stimulating factor (G-CSF), fibroblast growth factor 2 (FGF2), and vascular endothelial growth factor (VEGF) were lower (Figures 8(b)–8(d), 8(g), and 8(h)), in hAD-MSCs in the Rg1 group. However, the differences in the expressions of those cytokines were not significant between the Rg1 and control groups (*P* > 0.05, Figure 8).

To further confirm whether Rg1 can promote the expression and secretion of IGF-I in hAD-MSCs, ELISA was performed. It was found that the protein secretion level of IGF-I was significantly higher in hAD-MSCs in the Rg1 group than in the control group (*P* < 0.01, respectively; Figure 8(i)).

These results demonstrate that Rg1 may promote the expression and secretion of IGF-I in hAD-MSCs.

## 4. Discussion

This study shows that proper concentration of Rg1 can promote the viability, proliferation, and paracrine and relieve the senescence of hAD-MSCs. Rg1 may induce cell cycle progression and further promote the proliferation of hAD-MSCs through the upregulation of the expressions of CDKs and cyclins in hAD-MSCs. PI3K/Akt signaling pathway may be the upstream signaling of cyclins and CDKs for the mediation of Rg1-induced hAD-MSC proliferation. The protective effect of Rg1 on the senescence of hAD-MSCs may be achieved via the downregulation of p16^INK4A^ and p53/p21^CIP1^ pathway.

In the study, cells were isolated from human amnions, which were identified as hAD-MSCs by our previous published protocols [17]. Both our and other researches have proven that hAD-MSCs not only have the features of MSCs but also have unique merits for clinical utility [17, 36, 37], and hAD-MSCs represent a promising seed cell for regenerative medicine and clinical applications, which are worthy of further research.

Appropriate concentrations of Rg1 can benefit the viability of cells, while overdosages can cause toxicity to cells [38, 39]. Thus, the effects of Rg1 with different concentrations on the viability of hAD-MSCs were firstly researched in this study. It was found that Rg1 with the concentrations from 10 *μ*g/mL to 40 *μ*g/mL can significantly promote hAD-MSC viability, and the minimum effective concentration of Rg1 was selected for the subsequent experiments.

If MSCs were prepared as drugs for clinical use in the future, sufficient amounts of purified MSCs must be obtained [40, 41]. However, the number of MSCs gotten from tissues is mostly limited, which necessarily needs efficient expansion *in vitr*o [2, 42]. Although the number of hAD-MSCs obtained from human amnions and the proliferation rates of hAD-MSCs is relatively high [6–9], amnions are limited. Moreover, the decrease of MSC proliferation potency during *in vitro* culture and passaging is still a challenge of MSC-based therapy [43]. Thus, exploration of methods to promote hAD-MSC proliferation is still necessary. Gu et al. found that Rg1 can promote the proliferation of mouse BM-MSCs [25]. Xu et al. found that Rg1 from 10 to 100 *μ*g/mL can promote the proliferation of MSCs from human adipose tissue with obvious positive dose dependence [44]. We also found that Rg1 may promote cell cycle progression from G0/G1 to S and G2/M phases and facilitate the proliferation of hAD-MSCs. The results demonstrate that Rg1 may be a potent inducer of hAD-MSC proliferation.

Cell proliferation is the process whereby cells reproduce themselves by growing and then dividing into two equal copies. As the cell cycle gradually enters S and G2/M phases from G0/G1 phase, cell proliferation is finally fulfilled. To further explore the mechanisms of Rg1 on the proliferation of hAD-MSCs, regulatory proteins of cell cycle, cyclin D1, CDK4, cyclin E1 and CDK2, and PI3K/Akt signaling pathway in Rg1-induced hAD-MSCs were detected in this study.

As is known, cell cycle progression is regulated by cyclins and CDKs [30]. Various combinations of CDKs and cyclins regulate the orderly progression through the cell cycle [30]. Cyclin/CDK complexes are central components of the cell cycle signaling system. Cyclin D is low in resting cells (G0) and is an early component of cell cycle signaling. The expression of cyclin D in G1 cell cycle acts as the primary sensors of mitogens [45, 46]. The cell cycle is driven by the waves of cyclin formation that begin when mitogens activate the transcription of cyclin D. Cyclin D controls of G1 progression [30]. As the level of cyclin D rises, it combines with CDK4 to form an active complex which phosphorylates target proteins and in turn leads to the activation of cyclin E [17]. The increase of cyclin E level in cell cycle follows the rise of cyclin D during G1. Cyclin E pairs up with CDK2 and controls G1 progression and DNA synthesis (S phase). G1/S transition is essential for cell cycle progression [29]. Towards the end of G1, there is a restriction point, which marks the point where the cell becomes irreversibly committed to traverse the rest of the cell cycle [29]. The G1-to-S-phase transition is regulated by cyclin D/CDK4 and cyclin E/CDK2 complexes during the cell cycle [31]. In our study, we found that Rg1 upregulated the expressions of cyclin D1, cyclin E1, CDK4, and CDK2; induced cell cycle progression from G0/G1 into S and G2/M phases; and significantly promoted the proliferation of hAD-MSCs *in vitro*. These results demonstrate that Rg1 might promote cell cycle progression and cell proliferation by regulating the expressions of cyclins and CDKs in hAD-MSCs. However, the mechanisms by which Rg1 influences the expression of those regulatory proteins of cell cycle remain unclear.

The proliferative and antiproliferative signaling pathways interface with the cell cycle through controlling the activities of the cyclin/CDK complexes [17, 32]. PI3K/Akt signaling pathway is an important signaling to regulate cell cycle progression and boost cell proliferation and survival [32, 33]. PI3K signaling seems to be required for many mitogens in the G1-to-S phase transition of the cell cycle, which contributes to the build-up of cyclin D via increasing the stability and expression of the cyclin D mRNA [31]. Klippel et al. [31] found that the activation of PI3K was sufficient to promote G1 phase to S phase of the cell cycle and induce cell cycle progression within several hours by activating G1- and G1/S-phase cyclin/CDK complexes (cyclin D/CDK4 and cyclin E/CDK2) and for the induction of DNA synthesis. Akt is regarded as a major downstream effector molecule of PI3K. Activation of PI3K/Akt signaling pathway mediates cell cycle progression by inactivating the inhibitors of CDKs and activating CDK2 and CDK4, which facilitates G1-to-S-phase transition [17, 31, 32]. Studies have proved that PI3K/AKT signaling pathway can induce the expressions of cyclins and CDKs and promote cell proliferation [47, 48]. In our study, we found that Rg1 activated PI3K/AKT signaling pathway and synchronously upregulated the expressions of cyclin D1, cyclin E1, CDK4, and CDK2 in hAD-MSCs, which further promoted the cell cycle progression from G0/G1 phase into S and G2/M phases and the proliferation of hAD-MSCs. Moreover, the inhibition of PI3K/AKT signaling synchronously significantly downregulated the expressions of cyclin D1, cyclin E1, CDK4, and CDK2 in Rg1-induced hAD-MSCs, which in turn inhibited the cell cycle progression from G0/G1 phase into S and G2/M phases and the proliferation of hAD-MSCs induced by Rg1. These results demonstrate that Rg1 can activate PI3K/AKT signaling pathway in hAD-MSCs. CDKs and cyclins might be downstream molecules regulated by PI3K/AKT signaling pathway in Rg1-induced proliferation of hAD-MSCs. It is highly possible that PI3K/AKT signaling pathway is involved in the promotive effect of Rg1 on the proliferation of hAD-MSCs.

According to the combination of modern stem cell theory and “qi and blood” theory of traditional Chinese medicine, Rg1 might be an important drug to regulate the senescence of stem cells [28]. Xiang et al. [49] found that Rg1 regulated Wnt/*β*-catenin signaling pathway to delay the senescence of neural stem cells. Wang et al. [23] found that Rg1 can reduce the expression of senescence markers and effectively alleviate the senescence of mouse BM-MSCs via nuclear factor E2-related factor 2 (NRF2) and PI3K/Akt signaling. In this study, the specific method for senescence assay, SA-*β*-Gal staining, was conducted to detect the effects of Rg1 on the senescence of hAD-MSCs. It was demonstrated that Rg1 can alleviate the senescence of hAD-MSCs. To further explore the mechanisms of this process, two main senescence-related signaling pathways associated with DNA damage, p16^INK4A^ and p53/p21^CIP1^, which lead to cell cycle arrest and MSC senescence [34], were detected. During cellular senescence, the expression levels of p53, p21^CIP1^, and p16^INK4A^ were shown to be upregulated both *in vivo* and *in vitro* [34, 50]. Besides, inhibiting p21^CIP1^, p53, or p16^INK4A^ may also reduce the number of senescent MSCs and restore their proliferation ability [34, 51]. The senescent state is primarily characterized by durable cell cycle arrest [34]. Activation of CDK inhibitors, p16^INK4A^ and p21^CIP1^, is essential for senescence associated growth arrest, which antagonizes CDK to block cell cycle progression [34]. Various stresses acting on the p53 surveillance system can direct cells towards senescence. The activation of p53 can strongly increase the expression of p21^CIP1^ and trigger the senescence of stem cells [52–54]. The activation of p21^CIP1^ inhibits CDK2 and prevents CDK2-mediated inactivation of retinoblastoma (RB), which thereby enables RB to retain function and keep suppressing the E2 transcription factor (E2F), a key regulator of genes needed for cell growth control and proliferation [55, 56], eventually leading to cell cycle arrest in G1 phase and prevention of reentry [57, 58]. Similarly, p16^INK4a^ can inhibit CDK4 and prevent CDK4-mediated inactivation of RB to block cell cycle progression in G1 phase [34]. This mechanism can act either alone or in combination with the p53/p21^CIP1^ pathway [59]. It seems that p21^CIP1^ is often upregulated first and p16^Ink4a^ later, possibly representing distinct phases on the path from early to full senescence [59, 60]. The p14^ARF^ protein links the p16^INK4a^ pathway and p53/p21^CIP1^ pathway, which is also encoded by the INK4 locus and inhibits p53 degradation, thus favoring senescence [34]. In our study, D-gal was used to establish hAD-MSC aging models *in vitro*. It was found that D-gal significantly induced the expressions of p16^INK4a^, p14^ARF^, p21^CIP1^, and p53 in hAD-MSCs in the D-gal group, and Rg1 significantly reduced the elevated expressions of those senescence markers induced by D-gal in hAD-MSCs in the Rg1+D-gal group. Thus, we speculate that Rg1 might exert its protective effect against hAD-MSC senescence by downregulating the p16^INK4A^ and p53/p21^CIP1^ pathways.

Cellular senescence can be defined as a stable arrest of the cell cycle in G1 phase coupled to stereotyped phenotypic changes [61]. The G1-to-S-phase transition is regulated by cyclin D/CDK4 and cyclin E/CDK2 complexes during the cell cycle [31]. Thus, in our study, the expressions of CDK2, CDK4, cyclin D1, and cyclin E1 were also detected in normal, senescent, and Rg1-treated hAD-MSCs. It was found that the expressions of cyclin D1, cyclin E1, and CDK4 were significantly decreased in senescent hAD-MSCs after D-gal treatment in the D-gal group, while the expressions of cyclin D1, cyclin E1, and CDK4 were significantly increased by Rg1 treatment in senescent hAD-MSCs in the Rg1+D-gal group. These results also support that Rg1 may promote cell cycle progression and inhibit senescence of hAD-MSCs. Rg1 might be used as an adjuvant drug to alleviate the senescence of MSCs for MSC expansion *in vitro* and MSC therapy for diseases.

Previous studies have shown that MSCs can secrete a variety of cytokines, such as IL-1, IL-6, IL-10, FGF2, VEGF, HGF, G-CSF, and IGF-I, in a paracrine or autocrine manner [7, 35]. Many studies have shown that MSC secretome is primarily responsible for the benefits of MSC transplantation in repairing injury tissue [27, 62]. Our previous studies have also demonstrated that the ovarian function of premature ovarian insufficiency (POI) induced by chemotherapy in rats can be improved by hAD-MSC transplantation, and the mechanism is at least partly through the paracrine pathway of hAD-MSCs [7]. Our studies have proven that hAD-MSCs can secrete VEGF, FGF2, HGF, and IGF-I, and the presence of a paracrine mechanism accounting for hAD-MSC-mediated recovery of ovarian function in rats with chemotherapy-induced POI might be attributed to these growth factors secreted by hAD-MSCs [7]. A study found that Rg1 can enhance paracrine of BM-MSCs, which provides a novel way for maximizing the paracrine effects of MSCs [27]. In this study, it was found that Rg1 significantly promoted the expression and secretion of IGF-I in hAD-MSCs. IGF-I is an important growth and survival factors. IGF-I acts as a stimulator of cell proliferation and an inhibitor of cell apoptosis, which might be conducive to the repair of injury tissue [7, 63, 64]. The results suggest that Rg1 might be an attractive candidate to promote the therapeutic efficacy of hAD-MSC transplantation in the treatment of diseases.

Several studies showed that Rg1 can inhibit the apoptosis of BM-MSCs induced by the stimuli of hypoxia-reoxygenation [24], ischemia [65], and hydrogen peroxide [26]. We found that Rg1 can reduce the apoptosis of hAD-MSCs to an extent. However, the difference was not significant. The results are not consistent with the studies mentioned above [24, 26, 65]. We consider that the effects of Rg1 on the apoptosis of MSCs might vary with different proapoptotic factors, Rg1 concentrations, Rg1 treatment protocols, and derivation of stem cells, and much more work is needed to further define them in our subsequent experiments.

In this study, it was shown that Rg1 can significantly promote the proliferation and relieve the senescence of hAD-MSCs, which is consistent with its efficacy in mouse and human BM-MSCs [2, 23, 25, 28]. We speculate that Rg1 treatment might effectively regulate the proliferation and senescence of MSCs from different sources. However, this speculation needs more research and proof to confirm it. In addition, there are several limitations in this study. First, studies have shown that there are interdonor variability and scalability associated with the primary donor-derived MSCs [4, 11, 12], which might exhibit distinct biological properties and influence the results of our experiments. Second, in this study, the minimum effective concentration of Rg1 (10 *μ*g/mL) for hAD-MSC viability was selected for the subsequent experiments, which might be not the most appropriate concentration to improve all the biological behavior, such as apoptosis and migration, of hAD-MSCs. Third, we only discerned that PI3K/Akt signaling pathway may be the upstream signaling of cyclins and CDKs for the mediation of Rg1-induced hAD-MSC proliferation. However, the precise mediation mechanisms between them are still unclear. Therefore, in future study, hAD-MSCs should be manufactured under a rigorous quality control system, and further research will be done to explore and solve the problems mentioned above.

## 5. Conclusions

In conclusion, this study demonstrates that proper concentration of Rg1 is a favorable factor to promote the biological behavior of hAD-MSCs, which can promote the viability, proliferation, and paracrine and relieve the senescence of hAD-MSCs. PI3K/AKT signaling pathway is involved in the promotive effect of Rg1 on hAD-MSC proliferation. The protective effect of Rg1 on the senescence of hAD-MSCs may be achieved via the downregulation of p16^INK4A^ and p53/p21^CIP1^ pathway. Rg1 might show a promising application prospect with regard to the regulation of hAD-MSCs to promote the therapeutic efficacy of hAD-MSC transplantation for diseases.

## Figures and Tables

**Figure 1:** Effects of ginsenoside Rg1 on the viability of hAD-MSCs. (a–c) Morphology of hAD-MSCs ((a) ×40, (b) ×100, (c) ×200). (d–o) hAD-MSCs were able to differentiate into osteoblasts (d, f), adipocytes (h, j), and chondroblasts (l, n). The osteogenic differentiation of hAD-MSCs was verified by alizarin red S, and abundant calcium deposits stained with red were visualized (e, g). The adipogenic differentiation of hAD-MSCs was verified by oil red O staining, and red lipid vacuoles were visualized in the cytoplasm (i, k). The chondrogenic differentiation of hAD-MSCs was verified by alcian blue, and cartilage-specific proteoglycans stained with blue were visualized (m, o). (p) The molecular structure of ginsenoside Rg1. (q) The effects of Rg1 with different concentrations on the viability of hAD-MSCs were detected by CCK-8 assay. Optical density (OD) values at 450 nm of each concentration at 24 and 48 h after Rg1 treatment were shown (*n* = 6). Images of (d), (e), (h), (i), (l), and (m) were taken at 100x magnification, while (f), (g), (j), (k), (n), and (o) were taken at 200x. Representative images are shown. Scale bars = 100 *μ*m; Scale bars = 200 *μ*m. NS: not significant, ^∗^*P* < 0.05 and ^∗∗^*P* < 0.01.

**Figure 2:** Effects of ginsenoside Rg1 on the proliferation of hAD-MSCs. (a, b) The cell cycle phase distribution of the control and Rg1 groups was analyzed (a) and compared (b) by flow cytometry (*n* = 3). A representative image of three independent experiments is shown in each group. (c, d) The hAD-MSC proliferation rates of the control and Rg1 groups were tested (c) and compared (d) by EdU incorporation assay (100x) (*n* = 6). Representative images are shown. Scale bars = 100 *μ*m. (e) The growth curves of hAD-MSCs were detected using CCK-8 assay in the control and Rg1 groups (*n* = 6). ^∗^*P* < 0.05 and ^∗∗^*P* < 0.01.

**Figure 3:** Effects of ginsenoside Rg1 on the PI3K/AKT signaling pathway and expressions of cyclins and CDKs in hAD-MSCs. (a, b) The expressions of Akt, phospho-Akt, cyclin D1, cyclin E1, CDK2, and CDK4 in hAD-MSCs were analyzed (a) and compared (b) by western blot after pretreatment of hAD-MSCs with or without LY294002 for 1 h followed by the treatment with or without Rg1 in the control, Rg1, Rg1+LY294002, and LY294002 groups. ^∗^*P* < 0.05 and ^∗∗^*P* < 0.01.

**Figure 4:** Effects of ginsenoside Rg1 on the cell cycle phase distribution and proliferation of hAD-MSCs after blocking the PI3K/AKT signaling. (a, b) The cell cycle phase distribution of hAD-MSCs was detected (a) and compared (b) by flow cytometry after pretreatment of hAD-MSCs with or without LY294002 for 1 h followed by the treatment with or without Rg1 in the control, Rg1, Rg1+LY294002, and LY294002 groups (*n* = 3). (c–e) The proliferation of hAD-MSCs was detected and compared by CCK-8 (c) and EdU incorporation (d, e) assays after pretreatment of hAD-MSCs with or without LY294002 for 1 h followed by the treatment with or without Rg1 in the control, Rg1, Rg1+LY294002, and LY294002 groups (100x) (*n* = 6). A representative sample of three independent experiments is shown. Scale bars = 100 *μ*m. ^∗^*P* < 0.05 and ^∗∗^*P* < 0.01.

**Figure 5:** Effects of ginsenoside Rg1 on the apoptosis of hAD-MSCs. (a) The effects of D-gal with different concentrations on the viability of hAD-MSCs were detected using CCK-8 assay. Optical density (OD) values at 450 nm of each concentration at 24 and 48 h after D-gal treatment were shown (*n* = 6). (b) The morphology of hAD-MSCs in the control, Rg1, D-gal, and Rg1+D-gal groups (×100). (c, d) The hAD-MSC apoptosis rates in the control, Rg1, D-gal, and Rg1+D-gal groups were analyzed (c) and compared (d) by flow cytometry (*n* = 3). A representative image of three independent experiments is shown in each group. Scale bars = 200 *μ*m. NS: not significant, ^∗^*P* < 0.05 and ^∗∗^*P* < 0.01.

**Figure 6:** Effects of ginsenoside Rg1 on the senescence of hAD-MSCs. (a) Senescent cells were detected by SA-*β*-Gal staining in the control, D-gal, Rg1, and Rg1+D-gal groups (×100). (b) hAD-MSC senescence rates were compared in the control, D-gal, Rg1, and Rg1+D-gal groups. (c, d) The expressions of cyclin D1, cyclin E1, CDK2, CDK4, p14^ARF^, p21^CIP1^, p53, and p16^INK4a^ in hAD-MSCs were analyzed (c) and compared (d) by western blot in the control, D-gal, Rg1, and Rg1+D-gal groups. Representative images are shown. The red arrow indicates senescent hAD-MSCs stained with blue. Scale bars = 100 *μ*m. ^∗^*P* < 0.05 and ^∗∗^*P* < 0.01.

**Figure 7:** Effects of ginsenoside Rg1 on the migration of hAD-MSCs. (a) The migration of hAD-MSCs was tested by wound healing assay at 0, 12, and 24 h after Rg1 treatment *in vitro*, in the control, and Rg1 groups (100×). (b) The area-covered ratio of migration cells (ACRMC), which was defined as (covered area/scratched area) × 100%, was compared between the control and Rg1 groups (*n* = 3). Scratched areas and uncovered areas of hAD-MSCs were highlighted with red lines. Representative images are shown. Scale bars = 200 *μ*m. NS: not significant, ^∗^*P* < 0.05 and ^∗∗^*P* < 0.01.

**Figure 8:** Effects of ginsenoside Rg1 on the paracrine of hAD-MSCs. (a–h) The relative mRNA expression levels of HGF (a), FGF2 (b), G-CSF (c), VEGF (d), IGF-I (e), IL-10 (f), IL-6 (g), and IL-1*β* (h) in hAD-MSCs in the control and Rg1 groups were detected and compared by RT-qPCR. (i) The levels of IGF-I secreted by hAD-MSCs in the cell supernatant in the control and Rg1 groups were detected by ELISA. NS: not significant, ^∗^*P* < 0.05 and ^∗∗^*P* < 0.01.

**Table 1:** Primer sequences for PCR.

Gene	Primer sequence 5′→3′	Amplification	Accession no.
*G-CSF*	GCTCGGACACTCTCTGGGCATC	235 bp	NM_000759.4
	GGCCATTCCCAGTTCTTCCATC		
*HGF*	GCCGAGGCCATGGTGCTATAC	148 bp	NM_000601.6
	GCCCCTGTAGCCTTCTCCTTGAC		
*IGF-I*	GGTGGATGCTCTTCAGTTCGTGTG	155 bp	NM_001111283.3
	CGCAATACATCTCCAGCCTCCTTAG		
*VEGF*	GGGGCTGCTGCAATGACGAG	227 bp	NM_001025366.3
	CCGGGATTTCTTGCGCTTTC		
*FGF2*	CGCCAGGTCATTGAGATCCATC	143 bp	NM_002006.5
	TTCGGCAACAGCACACAAATCC		
*IL-1β*	GCGGCATCCAGCTACGAATCTC	247 bp	NM_000576.3
	TCCCGGAGCGTGCAGTTCAG		
*IL-6*	CCCCACACAGACAGCCACTCAC	131 bp	NM_000600.5
	TGCCTCTTTGCTGCTTTCACAC		
*IL-10*	AAAGGAGTCCTTGCTGGAGG	236 bp	NM_000572.3
	CATTCTTCACCTGCTCCACG		
*β-Actin*	ACCCCGTGCTGCTGACCGAG TCCCGGCCAGCCAGGTCCA	250 bp	NM_001101.5

G-CSF: granulocyte-colony stimulating factor; HGF: hepatocyte growth factor; IGF-1: insulin-like growth factor-1; VEGF: vascular endothelial growth factor; FGF2: fibroblast growth factor 2; IL-1*β*: interleukin-1*β*; IL-6: interleukin-6; IL-10: interleukin-10.

## Data Availability

The data used in this study are available from the corresponding author upon request.
